# Performance Assessment of Classification Algorithms on Early Detection of Liver Syndrome

**DOI:** 10.1155/2020/6680002

**Published:** 2020-12-12

**Authors:** Rashid Naseem, Bilal Khan, Muhammad Arif Shah, Karzan Wakil, Atif Khan, Wael Alosaimi, M. Irfan Uddin, Badar Alouffi

**Affiliations:** ^1^Department of IT and Computer Science, Pak-Austria Fachhochschule Institute of Applied Sciences and Technology, Haripur, Pakistan; ^2^Department of Computer Science, City University of Science and Information Technology, Peshawar, Pakistan; ^3^Research Center, Sulaimani Polytechnic University, Sulaimani 46001 Kurdistan Region, Sulaymaniyah, Iraq; ^4^Department of Computer Science, Islamia College Peshawar, Peshawar, KP, Pakistan; ^5^Department of Information Technology, College of Computers and Information Technology, Taif University, P.O.Box 11099, Taif 21944, Saudi Arabia; ^6^Institute of Computing, Kohat University of Science and Technology, Kohat 26000, Pakistan; ^7^Department of Computer Science, College of Computers and Information Technology, Taif University, P.O.Box 1109, Taif 21944, Saudi Arabia

## Abstract

In the recent era, a liver syndrome that causes any damage in life capacity is exceptionally normal everywhere throughout the world. It has been found that liver disease is exposed more in young people as a comparison with other aged people. At the point when liver capacity ends up, life endures just up to 1 or 2 days scarcely, and it is very hard to predict such illness in the early stage. Researchers are trying to project a model for early prediction of liver disease utilizing various machine learning approaches. However, this study compares ten classifiers including A1DE, NB, MLP, SVM, KNN, CHIRP, CDT, Forest-PA, J48, and RF to find the optimal solution for early and accurate prediction of liver disease. The datasets utilized in this study are taken from the UCI ML repository and the GitHub repository. The outcomes are assessed via RMSE, RRSE, recall, specificity, precision, G-measure, F-measure, MCC, and accuracy. The exploratory outcomes show a better consequence of RF utilizing the UCI dataset. Assessing RF using RMSE and RRSE, the outcomes are 0.4328 and 87.6766, while the accuracy of RF is 72.1739% that is also better than other employed classifiers. However, utilizing the GitHub dataset, SVM beats other employed techniques in terms of increasing accuracy up to 71.3551%. Moreover, the comprehensive outcomes of this exploration can be utilized as a reference point for further research studies that slight assertion concerning the enhancement in extrapolation through any new technique, model, or framework can be benchmarked and confirmed.

## 1. Introduction

The liver is well-thought-out to be one of the central organs in any living body with fundamental functions such as processing leftover products, generating enzymes, and eliminating exhausted tissues or cells [1]. We can stay alive merely a couple of days if our liver shuts down. Fortunately, the liver can continue its role even when up to 75% of it is contaminated or removed. This is due to its astonishing capability to produce new liver tissues from fine fettle liver cells that quiet exist [2]. It shows a significant role in several bodily functions such as protein creation and blood clotting to glucose (sugar), cholesterol, and iron metabolism. It has a range of functions, comprising eliminating toxins from the body, and is crucial for survival [3, 4]. The harm of these functions can reason to momentous destruction to the body. Once the liver is diseased with a virus, injured by chemicals, or under attack from its immune system, the elementary hazard is similar; that is, the liver will become so spoiled that it can no lengthier retain an individual alive [3, 5]. According to World Health Organization (WHO) and World Gastroenterology Organization (WGO), 35 million individuals pass away due to chronic diseases, and liver failure is one of the apprehensive diseases stated [6, 7]. It is further stated that more than 50 million grown-ups will be affected with chronic liver disease (CLD), and it requests for instantaneous responsiveness for actions in a conference held in Paris that deliberated the shocking drifts of liver disease worldwide [1, 8]. Moreover, agreeing to the current figures, 25 million US residents are pretentious by the liver or biliary ailment, and out of these, 50% populace have no symptoms. In the United Kingdom, nearly 25% of death due to liver disease is from extreme alcohol drinking [9].

## 2. Foremost Reasons for Liver Disease

As soon as the liver becomes diseased, it can ground severe destruction to our health. There can be numerous equipment and health conditions that can naively reason for liver damage [10–12].

### 2.1. Alcohol

Dense alcohol drinking is the utmost collective reason for liver damage. Once individuals drink alcohol, the liver becomes distracted from its other functions and provides attention mostly on converting alcohol into a smaller amount of toxic form.

### 2.2. Obesity

People who are fat have the leftover quantity of body obese which inclines to accrue nearby the liver causing fatty liver disease (FLD).

### 2.3. Diabetes

Devising diabetes upturns the hazard of liver disease by 50 percent. Increased level of compelling insulin results in FLD.

## 3. Common Liver Disorder

### 3.1. Hepatitis

It is an ailment produced by a virus feast due to manure pollution or direct interaction with the septic bloody fluids [5].

### 3.2. Cirrhosis

It is the utmost severe liver disease that happens when normal liver cells are swapped by mutilation tissue as the CLD [4, 13].

### 3.3. Liver Cancer

The danger of consuming liver cancer is higher for individuals who have cirrhosis and another type of hepatitis [12].

In the current era, we have been confronted with a cumulative amount of records kept in several societies such as hospitals, universities, and banks that inspire us to discover an approach to mine information from this huge number of records and to proficiently use them, especially in the healthcare organizations. In the recent era, researchers are focusing on using data from healthcare organisations for early and accurate prediction of syndromes. Nowadays, data mining (DM) and machine learning (ML) become elementary in healthcare due to its approaches, e.g., classification, clustering, and association rule mining, for determining repeated patterns pragmatic for disease extrapolation on medical data [6, 14].

In the early past, researchers have used different ML techniques for the early and accurate prediction of liver as well as some other diseases. Hassoon et al. [15] used genetic algorithm (GA) for the early prediction of liver syndromes. They have evaluated their model based on accuracy rate, specificity, sensitivity, precision, F1, and false-positive rate. The outcomes are compared with Boosted C5.0, and the results show the best performance of GA with a higher accuracy of 92.23%. Research in [16] focused on liver syndrome by taking ten significant features and using Decision Tree (DT) approaches, Naïve Bayes (NB), and NBTree (NBT) techniques to classify the syndrome's indications. Lastly, they perceived that the NBT technique is most precise than NB for emancipating rules. In [14], for forecasting liver syndrome, they used NB and support vector machine (SVM) for classification, and as a final point, they originate that SVM has better concert and accuracy in liver syndrome classification. A new approach of classification that will relieve suitable and interpretable rules is recursive-rule extraction (Re-RX) which is utilized in [17] to extract more and effective rules for the liver syndrome analysis.

In [18], for discovering the actual rules on liver syndrome analysis, C4.5 procedure smears as one of the well-known DT procedures in classification. Like, in [18, 19], C4.5 technique is used, and the researchers strained to utilize the technique for identifying liver syndrome. We can comprehend that C4.5 has a virtuous response on various types of disease analysis such as diabetes [20] and breast cancer [21]. Likewise, in [6], there is an assessment among C5.0 and CHAID techniques on the liver syndrome, and lastly, they found out that boosted C5.0 has a better response on discovering effectual rules. Boosting is a technique used in the C5.0 technique to increase this version over C4.5. Similarly, it increases the accuracy rate and the runtime of the algorithm [6].

However, the persistence of this study is the performance analysis of various ML classification algorithms on the liver disease dataset taken from UCI ML repository and GitHub repository. The classification algorithms include average one dependency estimator (A1DE), multilayer perceptron (MLP), NB, K-nearest neighbour (KNN), SVM, composite hypercube on iterated random projection (CHIRP), credal decision tree (CDT), forest by penalizing attributes (Forest-PA), decision tree (J48), and random forest (RF). To evaluate the performance analysis of these classifiers, different performance assessment measures are utilized which embrace root relative squared error (RRSE), root mean squared error (RMSE), specificity, precision, recall, F-measure, G-measure, Matthew's correlation coefficient (MCC), and accuracy.

The rest of the paper is prepared as follows: Section 2 contains the methodology of this research that comprises further subsections of dataset description, performance assessment measures, and review of employed techniques.  Section 3 grants the experimental results and discussion, and Section 4 and Section 5, respectively, present the threats to validity and the overall conclusion of this research.

## 4. Methodology

This research aims to present the performance analysis of ML classification algorithms for liver disease prophecy on two different datasets occupied from GitHub and UCI ML repositories. The complete research is prepared via the procedure shown in Figure 1. After the selection of datasets, a preprocessing step is applied on each dataset for two main purposes: replacing the missing values and changing the class attribute from numerical to categorical due to some of the techniques that do not work on numerical class attributes. After all, when ML techniques are applied to each dataset, the outcomes are assessed using different assessment measures to show the better performance of an individual technique. For this, nine assessment measures, namely, RMSE [22–24], RRSE [25], specificity [26–28], precision [29–31], recall [27, 29, 32], F-measure [29, 30, 33], G-measure [22, 34], MCC [29, 35, 36], and accuracy [3, 37, 38], are utilized to assess the performance of ML classification algorithm going on liver datasets.

### 4.1. Datasets Description

Each dataset is consisting of some attributes along with a known output class. Respectively, datasets contain numerical data, while the total number of attributes and instances is different. There are two liver datasets utilized in this study. One is taken from the UCI ML repository (https://archive.ics.uci.edu/ml/datasets/liver+disorders), and the second is from the GitHub repository (https://github.com/SanikaVT/Liver-disease-prediction).  Table 1 presents the details of the attributes of the dataset taken from the UCI ML repository, whereas Table 2 presents the same for the dataset taken from the GitHub repository. The first dataset (taken from the UCI ML repository) comprises seven features in which the first five features are all blood examinations which are believed to be thoughtful to liver diseases that might arise from extreme alcohol feeding. There are a total of 345 records in this dataset amid these 345: 145 are liver patients, and the rest of 200 are nonliver patient's records. In the second dataset (taken from GitHub repository), eight features are all blood tests, which is supposed to be thoughtful to liver disorder. This dataset contains a total of 583 records. Among these records, 416 are the liver patients, while the rest 167 are nonliver patient's records.  Figure 2 shows the percentage of liver patients and nonliver patients in both datasets. In each dataset, the last attribute is known as a selector containing the value 1 or either 2. Value 1 represents that the person is a positive liver patient, whereas 2 shows the nonliver patients' records.  Figure 2 shows the number of liver patients and nonliver patients for each dataset.

### 4.2. Performance Measurement Parameters

Performance assessment of every model utilized is a significant part of any research study. A model may produce satisfactory results when it is assessed using standard assessment measures. However, in this study, two types of assessment measures are used in which some are utilized for evaluating error rate that includes RMSE [25, 39] and RRSE [25], while others are employed for the assessment of accuracy that comprises specificity [5, 40], precision [32, 41], recall [31, 42], F-measure [29, 36], G-measure [22, 34], MCC [29, 35, 36], and accuracy [3, 37, 38].  Table 3 shows the equation for calculating each assessment measure with equations, where |*y*_*i*_ − *y*| is the absolute error, *n* is the number of errors, *T*_*j*_ is the goal value for record *ji*, *P*_*ij*_ is the prediction rate by the particular model *I* for data *j* (out of *n* records), TP presents the true-positive classification, FN shows the false-negative classification, TN grants the true-negative classification, and FP is the rate of false-positive classifications.

## 5. Summarization of Employed Techniques

This subsection comprises a brief review of techniques employed in this research and contrasted with RF.

### 5.1. Average One Dependency Estimator

A1DE is a probabilistic technique used for mostly classification problems. It succeeds in extreme precise classification by averaging inclusive of a minor space of different NB-like models that have punier independence suppositions than NB. A1DE was designed to address the attribute-independence issues of a popular NB technique. It was designed to address the attribute-independence issues of the prevalent NB classifier [43].

### 5.2. Naïve Bayes

NB is known as the kinfolk of modest probabilistic classifiers grounded on Bayes hypothesis with individuality suppositions amid the predictors [44, 45]. NB model is precise simple to construct and can be executed for any dataset containing a large amount of data. The posterior probability *P*(*c*/*x*) is taken as of *P*(*c*), *P*(*x*), and *P*(*x*/*c*). The consequence of the rate of a predictor *(x)* on assumed class *(c)* is autonomous of the rate of other predictors.

### 5.3. Multilayer Perceptron

MLPs are deliberated as the utmost momentous classes of the neural network comprising an input layer, at least one hidden layer, and an output layer [46, 47]. The techniques behind the neural network are that when data are accessible as the input layer, the network neurons start calculation in the sequential layer till an output value is gained at each of the output neurons. A threshold node is moreover added to the input layer which identifies the weight function [48].

### 5.4. Support Vector Machine

It is a managed learning technique that has several uses in the ground of classification, biophotonics, and pattern recognition [22]. Firstly, it was developed for binary classification; however, it can also be used for multiple classes [41]. In binary classification, SVM classifies data by finding the best hyperplane that separates all data points in one class from those in the other class. In that case, if data are linearly inseparable, a mathematical function is utilized to transmute the records to an advanced dimensional space such that it possibly will grow into linear divisible in the new space [27].

### 5.5. K-Nearest Neighbour

KNN is a supervised learning technique where the preparation of features attributes to forecast the class of new test data. KNN classifies the first-hand data grounded on leased space from the new records to the *k*-nearest neighbors [9]. The nearest distance can be found using different distance functions like Manhattan distance (MD), Euclidean distance (ED), and Minkowski distance (MkD) [49].

### 5.6. Composite Hypercube on Iterated Random Projection

It is a reiterative module of three levels: anticipating, binning, and covering, which projected to a defrayal with the thorn in your side of computational unpredictability, dimensionality, and nonlinear recognisability [50]. CHIRP is not the cascading of diverse techniques, also not the enhancement or modification of attractive techniques; it utilizes new packaging techniques. The exactness of this technique usually utilized unbiased datasets and leaves behind the accuracy of contestants. The CHIRP uses computationally convincing ways to deal with accumulating 2D predictions and sets of quadrangular regions on those predictions that include valuations from a separable crowd of data. CHIRP categorizes these crowds of forecasts and segments them into a final incline for the accumulation of new data estimation [51].

### 5.7. Credal Decision Tree

CDT is a technique to design classifiers grounded on inexact possibilities and improbability measures [52]. Throughout the creation procedure of a CDT, toward sidestep producing an also problematical decision tree, a new standard remained presented: stop once the overall improbability rises because of the splitting of the decision tree. The function utilized in the overall indecision dimension can be fleetingly articulated as in [53, 54].

### 5.8. Forest by Penalizing Attributes

Forest-PA uses bootstrap samples and penalized attributes. It purposes to construct a group of extremely precise decision trees by manipulating the strong point of entirely nonclass features presented in a dataset, not like certain current techniques that utilized a subgroup of the nonclass features. Next to a similar time to support robust assortment, Forest-PA enforces disadvantages (detrimental weights) en route for individual's features that contributed to happening on the newest tree to produce the consequent trees. Forest-PA moreover consumes a contrivance toward step-by-step rise loads from the features that have not been verified in the consequent tree(s) [55].

### 5.9. Decision Tree (J48)

This is the basic C4.5 Decision Tree (DT) used for classification problems [37]. It is the deviation of information gain (IG), usually utilized to stun the result of biasness. An attribute using a maximum gain ratio is nominated in direction to shape a tree as a dividing attribute. Gain ratio- (GR-) based DT performs well as compare to IG, in terms of accuracy [4].

### 5.10. Random Forest

RF produces a set of techniques that involve constructing an ensemble or so-termed as a forest of decision trees from a randomized variation in tree induction techniques [1]. RF works through forming a mass of decision trees at the preparation period and outputting the group in the approach of the group output by a single tree. It is deliberated as one of the utmost techniques which is extremely proficient for both classification and regression problems [56].

## 6. Experimental Results

This section comprises the experimental analysis of liver syndrome prophecy utilizing ten ML classifiers. For training and testing, 10-fold cross-validation is used which is a standard methodology for assessments [41]. The ML classifiers are evaluated on the dataset available online on the UCI ML repository and GitHub repository. The overall experimental analysis shows the error rates (achieved via RMSE and RRSE) as well as accuracy (succeeded through specificity, recall, precision, G-measure, F-measure, MCC, and accuracy). The experimental analysis is subdivided into two sections that are scenario 1 and scenario 2. Scenario 1 represents the outcomes of algorithms employed on dataset taken from the UCI ML repository, while scenario 2 represents the same on dataset taken from the GitHub repository.

### 6.1. Experimental Results: Scenario 1 (UCI Dataset)

Here, firstly, we discuss the experiments carried out to find the minimum error rate assessed by RMSE and RRSE achieved via each classifier. These results are given in Table 4 where the second column shows the list of employed classifiers while the third column and fourth column, respectively, represent the results of RMSE and RRSE. This table shows that RF outperforms other classifiers in terms of reducing error rates; the results are 0.4328 for RMSE and 87.6766 for RRSE. In the rest of the classifiers, MLP produces better results in reducing both RMSE and RRSE, and the results achieved are 0.4532 and 91.6375, respectively.

Table 5 shows the detail of correctly classified instances (CCIs) and incorrectly classified instances (ICIs) amid an overall of 345 instances. The greater CCI rates show the best performance of an individual classifier.  Table 6 represents the standings of confusion matrix (CM), while Table 7 represents the CM for all the assessments calculated throughout experimentations. There are binary classes in which predicting is promising, i.e., class 1 and class 2. Class 1 is also known as positive, while class 2 is known as negative. If we predict the existence of a disease, in the case, class 1 proceeds that the individual ensures the disease, while class 2 proceeds that the individual does not ought to the disease. Here, TP is the situation where the persistent as positive (they ought to the disease), and FP is likewise the condition of positive, but they ought no to the disease, which is known as type 1 error. FN illustrates the negative conditions, but they in fact ought to the disease which is called type 2 error. TN demonstrates a negative situation, which indicates that they ought not to the disease. The values of CM are employed in finding complete accuracy outcomes. In our case, these are specificity, recall, precision, G-measure, F-measure, MCC, and accuracy according to equations (see Table 3).

Table 8 signifies the assessed outcomes of specificity, precision, recall, F-measure, G-measure, MCC, and accuracy concerning each classifier. The values of each of these measures are calculated with help of CM (see Table 7). The best performance of each classifier assessed via every evaluation metric is mentioned in bold. This analysis shows that, by evaluating each classifier through specificity, F-measure, MCC, and accuracy, RF outperforms other classifiers and achieved better results. The details of according to these measures are presented in Figure 3 while Figure 4 presents the accuracy details. In the case of precision, NB results are better than the rest of the classifiers while on recall and G-measure, SVM outperforms other classifiers employed.  Figure 5 shows the percentage difference in terms of accuracy between RF and other employed classifiers. The difference is calculated via the following equation:

(1) $$\begin{array}{c} \text{percentage difference}=\;\frac{\left|v_{i}-v_{j}\right|}{\left(v_{i}+v_{j}/2\right)}{}^{*}100, \end{array}$$

where *v*_*i*_ and *v*_*j*_ are the values in which the difference is to be calculated.

Figure 4 illustrates that there is very little difference between RF and MLP and RF and CHIRP, which is 0.81% and 1.21%, respectively.

### 6.2. Experimental Results: Scenario 2 (GitHub Dataset)

Here, first, we discuss the experiment carried out to find the minimum error rate assessed by RMSE and RRSE achieved via an individual classifier. The outcomes are shown in Table 9 where the second column represents the list of employed classifiers while the third column and fourth column, respectively, represent the results of RMSE and RRSE. This table shows that RF outperforms other classifiers in terms of reducing error rates, and the results are 0.4225 for RMSE and 93.4416 for RRSE. Despite the classifiers, MLP outperforms other classifiers in terms of reducing the error rate. The results achieved via MLP are 0.4276 and 94.5776 in that order for RMSE and RRSE.

Table 10 presents the details of CCI and ICI among a total of 583 instances. The larger ICI rate shows the best performance of that classifier.  Table 11 represents the CM for all the assessments assessed throughout the experiments.

Table 12 signifies the outcome assessed via specificity, precision, recall, F-measure, G-measure, MCC, and accuracy. These outcomes show the best performance of three different classifiers for different assessment measures. According to these analyses, A1DE beats other classifiers in terms of better results of specificity and G-measure that are 0.4680 and 0.5934 accordingly. NB outperforms other techniques in terms of good results for recall and MCC that are 0.9540 and 0.3469, respectively. However, SVM outperforms other classifiers by increasing the rate of precision, F-measure, and accuracy. The results achieved are 1 for precision, 0.8328 for F-measure, and 71.3551% accuracy. These outcomes are illustrated in Figure 6, while Figure 7 represents the accuracy details of each classifier which shows the best performance of SVM. The accuracy difference between SVM and other classifiers is presented in Figure 8.

## 7. Results Discussion

This research focuses on the performance analysis of ten various and well-known ML classification algorithms on two different liver disease datasets taken from the UCI ML repository and GitHub repository. On both datasets, results, after the evaluation is different due to each dataset, contain different amounts of instances, attributes, dataset according to attributes, and, the most important, different amount (percentage) of affected and nonaffected patient records.  Table 13 shows the better performance of optimal classifiers on both datasets concerning each assessment measure. These analyses illustrate that, in terms of reducing the error rate on both datasets, RF outperforms other classifiers. Moreover, RF also outclasses additional employed techniques in rapports of increasing accuracy on the dataset in use from the UCI ML repository. This is because RF is an excessive classifier with high-dimensional data; meanwhile, we are at work with subsets of data. To succeed in the prediction using the trained RF, classifier desires to permit the test features through the information of each randomly generated tree [7, 57]. RFs agonize fewer overfitting to a specific dataset than simple trees. RFs were constructed via merging the forecasts of numerous trees that are trained in separation, which provide valuable internal assessments of strength, error, correlation, and variable prominence [29, 58]. However, on the UCI dataset, SVM produces better results for recall and G-measure assessment measures. On the contrary, on the dataset taken from the GitHub repository, SVM performs better in terms of increasing accuracy as well as precision and F-measure. The SVM is the progressive tool with thoroughgoing classification algorithms surrounded in statistical learning theory [14]. It utilizes a nonlinear mapping to recondition the exclusive training data keen on a higher dimension [59]. Conversely, on the same dataset, A1DE also performs better in terms of increasing the rate of specificity and G-measure while NB does the same for recall and MCC.

### 7.1. Model Preparation

A model for liver syndrome prophecy is proposed, evaluated, and validated to test and compare results of ten various ML classification algorithms including A1DE, NB, MLP, SVM, KNN, CHIRP, CDT, Forest-PA, J48, and RF, and as the results revealed that RF is best suitable classifier in the environment related to prediction of liver syndromes in rapports of both increasing accuracy and reducing error rate on the dataset occupied from UCI ML repository. However, on the dataset taken from GitHub repository, SVM is the optimal solution for increasing accuracy although RF is the best solution to reduce the error rates.

### 7.2. Objectives Accomplished

#### 7.2.1. Objective 1

It was to propose a model for liver syndrome prophecy that will help to increase the accuracy and reduce error rate in early prophecy.

#### 7.2.2. Objective 2

It was to compare the results of classification algorithms to achieve most optimal solution for early and accurate prediction of liver syndromes.

### 7.3. Threats to Validity

This section contains the effects that might anguish the cogency of this research work.

*Internal Validity.* The exploration of this research is grounded proceeding diverse and very familiar evaluation standards that are used in the past in various studies. Amid these standards, several techniques are used to assess the error rate while certain techniques were used to assess the accuracy. So, the treat can be that renewal of new evaluation standards as a replacement for utilized standards can decrease the accuracy. Furthermore, the techniques used in this exploration can be supplanted using several newest techniques or can be cascaded with each other that can harvest enhanced outcomes as compared to the employed techniques.

*External Validity.* This study piloted investigations on two datasets occupied from UCI ML and GitHub repositories. The threat to validity might rise due to the condition of relating the projected techniques in other existent data composed from the various medical organizations or replacing these datasets with some other datasets, which may distress the outcomes while growing the error rates. Likewise, the projected technique possibly will not be capable toward harvesting improved forecast in outcomes via certain additional datasets. Hence, this research concentrated on datasets available on UCI ML repository and GitHub repository to measure the performance of the employed techniques.

*Construct Validity.* In this research, diverse ML techniques remain benchmarked through each other, going on liver dataset occupied from UCI ML and GitHub repositories using several valuation measures. The assortment of techniques utilized in this study is on the center of their progressive characteristic above the other techniques that ought to be exploited by the canvassers in the last decades. However, it can be a threat if we put on some other new techniques, and the outcomes can be improved probably than the projected techniques. In addition, the increase or decrease in training or testing samples from the dataset has a significant impact on the error rate. Likewise, choosing a different number of folds during K-fold validation has a dramatic effect on the error rate. The newest evaluation standards can also produce improved outcomes that can beat current accomplished outcomes.

## 8. Conclusions

Liver diseases are rising on daily basis, and it is hard to foresee these ailments in the early premise. Researchers have utilized a large number of ML techniques to foresee such ailments in the initial stage, but still there is need to improve accuracy as well as reduce error rates in the projected models. However, in this study, ten different ML classifiers including A1DE, NB, MLP, SVM, KNN, CHIRP, CDT, Forest-PA, J48 and RF are benchmarked on two different liver disease datasets taken from UCI ML repository and GitHub repository. For the assessments of these classifiers, nine standard assessment standards are utilized which are RMSE, RRSE, specificity, recall, precision, G-measure, F-measure, MCC, and accuracy. The overall experiments in use on UCI ML repository dataset show the best performance of RF. RMSE and RRSE results of RF are 0.4328 and 87.6766 correspondingly, while accuracy is 72.1739%. Moreover, RF also performs better in terms of reducing error rate on the dataset from GitHub repository, and the achieved results are 0.4225 and 93.4416, respectively, for RMSE and RRSE. However, in terms of increasing accuracy on the GitHub repository dataset, SVM achieved a higher accuracy of 71.3551%.

### 8.1. The Major Contributions of This Research

  We associate the results of ten ML classifiers including A1DE, NB, MLP, SVM, KNN, CHIRP, CDT, Forest-PA, J48, and RF.
  We acquit a series of experiments on liver disease datasets accessible on UCI ML and GitHub repositories.
  To deliver vision into the experimental outcomes, evaluation is conceded out via RRSE, RMSE, specificity, recall, precision, G-measure, F-measure, MCC, and accuracy.

### 8.2. Significance Statement

In this study, we employed ten ML classifiers on two different liver disease datasets that are occupied from the UCI ML repository including 345 cases and GitHub repository enclosing 583 cases. The results of stated techniques have been compared with characterising the utmost accurate technique that conveys around categorizing the affected and nonaffected patients with less error rate and high accuracy. This study recommended the RF and SVM are the best techniques that can be employed by physicians so as to exterminate treatment and diagnostic errors.

## Figures and Tables

**Figure 1:** Methodology workflow diagram.

**Figure 2:** Number of liver patient and nonliver patient for each dataset: (a) UCI ML repository; (b) GitHub repository.

**Figure 3:** Specificity, precision, recall, F-measure, G-measure, and MCC analysis representation.

**Figure 4:** Accuracy achieved via each classifier.

**Figure 5:** Accuracy percentage difference between RF and other employed classifiers.

**Figure 6:** Specificity, recall, precision, MCC, F-measure, and G-measure analysis representation.

**Figure 7:** Accuracy representation.

**Figure 8:** Accuracy percentage difference between SVM and other employed classifiers.

**Table 1:** List of dataset attributes and descriptions taken from the UCI ML repository.

S. no.	Attribute	Value type	Normal value range	Description
1	MCV	Integer	75–95	Mean corpuscular volume
2	Alkphos	Integer	63–2110	Alkaline phosphatase
3	SGPT	Integer	10–2000	Alanine aminotransferase
4	SGOT	Integer	10–4929	Aspartate aminotransferase
5	GammaGT	Integer	12–64	Gamma-glutamyl transpeptidase
6	Drinks	Real	-	Number of half-pint equivalents of alcoholic beverages % drunk per day
7	Selector	Selector {1, 2}	-	Field used to split data into two sets

**Table 2:** List of dataset attributes and descriptions taken from the GitHub repository.

S. no.	Attribute	Value type	Normal value range	Description
1	Age	Integer	4–90 years	Age of the patient
2	Gander	Text	Male/female	Gander of the patient
3	TB	Integer	0.4–75	Total bilirubin
4	DB	Integer	0.1–19.7	Direct bilirubin
5	Alkphos	Integer	63–2110	Alkaline phosphatase
6	SGPT	Integer	10–2000	Alanine aminotransferase
7	SGOT	Integer	10–4929	Aspartate aminotransferase
8	TP	Integer	2.7–9.6	Total proteins
9	ALB	Integer	0.9–5.5	Albumin
10	A/G ratio	Integer	0.3–2.8	Albumin and globulin ratio
11	Selector {1, 2}	Integer	1–2	Field used to split data into two sets

**Table 3:** Performance assessment measures to evaluate the experimental results.

S. no.	Measure	Description and equation
1	RMSE	$\text{RMSE}=\;\sqrt{1/2\sum_{j=1}^{n}{\left(y_{i}-1\right)}^{2}}$
2	RRSE	$\text{RRSE}=\;\sqrt{\sum_{j=1}^{n}{\left(P_{ij}-T_{j}\right)}^{2}/\sum_{j=1}^{n}{\left(T_{j}-T\right)}^{2}}$
3	Specificity	Specificity=TN/FP+TN
4	Precision	Precision=TP/TP+FP
5	Recall	Recall=TP/TP+FN
6	F-measure	FM=2^*∗*^precision^*∗*^recall/precision+recall
7	G-measure	GM= 2^*∗*^recall^*∗*^specificity/recall+specificity
8	MCC	$\text{MCC}=\left(\text{TN}{}^{*}\text{TP}\right)-\left(\text{FN}{}^{*}\text{FP}\right)/\sqrt{\left(\text{FP}+\text{TP}\right)\left(\text{FN}+\text{TP}\right)\left(\text{TN}+\text{FP}\right)\left(\text{TN}+\text{FN}\right)}$
9	Accuracy	Accuracy= TP+TN/TP+TN+FP+FN

**Table 4:** RMSE and RRSE outcomes assessments.

S. no.	Classifier	RMSE	RRSE
1	A1DE	0.4995	101.1922
2	NB	0.5083	102.9673
3	MLP	0.4523	91.6375
4	SVM	0.6461	130.8811
5	KNN	0.6072	123.0036
6	CHIRP	0.5357	108.5209
7	CDT	0.5005	101.3988
8	Forest-PA	0.4563	92.4357
9	J48	0.5025	101.8061
10	RF	**0.4328**	**87.6766**

**Table 5:** Results of CCI and ICI achieved via each classifier.

S. no.	Technique	CCI	ICI
1	A1DE	194 (56.2%)	151 (43.8%)
2	NB	191 (55.4%)	154 (44.6%)
3	MLP	247 (71.6%)	98 (28.4%)
4	SVM	201 (58.3%)	144 (41.7%)
5	KNN	217 (62.9%)	128 (37.1%)
6	CHIRP	246 (71.3%)	99 (28.7%)
7	CDT	219 (63.5%)	126 (36.5%)
8	Forest-PA	241 (69.9%)	104 (30.1%)
9	J48	237 (68.7%)	108 (31.3%)
10	RF	249 (72.2%)	96 (27.8%)

**Table 6:** Terms of confusion matrix.

	Positive or class 1 (1)	Negative or class 2 (0)
Positive or class 1 (1)	True positive	False positive
Negative or class 2 (0)	False negative	True negative

**Table 7:** Confusion matrix for all classifiers.

S. no.	Technique	TP	FP	FN	TN
1	A1DE	33	112	39	161
2	NB	111	34	120	80
3	MLP	83	62	36	164
4	SVM	1	144	0	200
5	KNN	82	63	65	135
6	CHIRP	82	63	36	164
7	CDT	60	85	41	159
8	Forest-PA	74	71	33	167
9	J48	77	68	40	160
10	RF	90	55	41	159

**Table 8:** Outcomes assessed via specificity, recall, precision, G-measure, F-measure, MCC, and accuracy.

S. no.	Technique	Specificity	Precision	Recall	F-measure	G-measure	MCC	Accuracy
1	A1DE	0.5897	0.2276	0.4583	0.3041	0.5158	0.0396	56.2319
2	NB	0.7018	**0.7655**	0.4805	0.5904	0.5704	0.1737	55.3623
3	MLP	0.7257	0.5724	0.6975	0.6288	0.7113	0.4075	71.5942
4	SVM	0.5814	0.0069	**1**	0.0137	**0.7353**	0.0633	58.2609
5	KNN	0.6818	0.5655	0.5578	0.5616	0.6136	0.2401	62.8986
6	CHIRP	0.7225	0.5655	0.6949	0.6236	0.7084	0.4011	71.3043
7	CDT	0.6516	0.4138	0.5941	0.4878	0.6215	0.2265	63.4783
8	Forest-PA	0.7017	0.5103	0.6916	0.5873	0.6966	0.3685	69.8551
9	J48	0.7018	0.531	0.6581	0.5878	0.6792	0.3452	68.6957
10	RF	**0.743**	0.6207	0.687	**0.6522**	0.7139	**0.4228**	**72.1739**

**Table 9:** RMSE and RRSE outcomes assessments.

S. no.	Technique	RMSE	RRSE
1	A1DE	0.4479	99.074
2	NB	0.6541	144.6684
3	MLP	0.4276	94.5776
4	SVM	0.5352	118.3788
5	KNN	0.5976	132.1834
6	CHIRP	0.5432	120.1379
7	CDT	0.4492	99.3545
8	Forest-PA	0.4379	96.8574
9	J48	0.4797	106.1058
10	RF	**0.4225**	**93.4416**

**Table 10:** Results of CCI and ICI achieved via each classifier.

S. no.	Technique	CCI	ICI
1	A1DE	403 (69.1%)	180 (30.9%)
2	NB	325 (55.7%)	258 (44.3%)
3	MLP	398 (68.3%)	185 (31.7%)
4	SVM	416 (71.4%)	167 (28.6%)
5	KNN	374 (64.2%)	209 (35.8%)
6	CHIRP	411 (70.5%)	172 (29.5%)
7	CDT	403 (69.1%)	180 (30.9%)
8	Forest-PA	401 (68.8%)	182 (31.2%)
9	J48	402 (69%)	181 (31%)
10	RF	404 (69.3%)	179 (30.7%)

**Table 11:** Confusion matrix for all classifiers.

S. no.	Technique	TP	FP	FN	TN
1	A1DE	308	108	72	95
2	NB	166	250	8	159
3	MLP	351	65	120	47
4	SVM	416	0	167	0
5	KNN	297	119	90	77
6	CHIRP	368	48	124	43
7	CDT	367	49	131	36
8	Forest-PA	358	58	124	43
9	J48	345	71	110	57
10	RF	355	61	118	49

**Table 12:** Outcomes assessed via specificity, recall, precision, G-measure, F-measure, MCC, and accuracy.

S. no.	Technique	Specificity	Precision	Recall	F-measure	G-measure	MCC	Accuracy
1	A1DE	**0.4680**	0.7404	0.8105	0.7739	**0.5934**	0.2935	69.1252
2	NB	0.3886	0.399	**0.9540**	0.5627	0.5524	**0.3469**	55.7461
3	MLP	0.4196	0.8438	0.7452	0.7914	0.5369	0.1437	68.2676
4	SVM	#DIV/0!	**1**	0.7136	**0.8328**	#DIV/0!	#DIV/0!	**71.3551**
5	KNN	0.3929	0.7139	0.7674	0.7397	0.5197	0.1675	64.1509
6	CHIRP	0.4725	0.8846	0.748	0.8106	0.5792	0.177	70.4974
7	CDT	0.4235	0.8822	0.7369	0.8031	0.5379	0.1253	69.1252
8	Forest-PA	0.4257	0.8606	0.7427	0.7973	0.5412	0.141	68.7822
9	J48	0.4453	0.8293	0.7582	0.7922	0.5611	0.1864	68.9537
10	RF	0.4454	0.8534	0.7505	0.7987	0.5591	0.1696	69.2967

**Table 13:** Performance of optimal classifiers on datasets according to each assessment measures.

S. no.	Assessment measures	Dataset from UCI ML repository	Dataset from GitHub repository
1	RMSE	RF	RF
2	RRSE	RF	RF
3	Specificity	RF	A1DE
4	Precision	NB	SVM
5	Recall	SVM	NB
6	F-measure	RF	SVM
7	G-measure	SVM	A1DE
8	MCC	RF	NB
9	Accuracy	RF	SVM

## Data Availability

The data utilized for finding the outcomes of this research have been taken from UCI ML and GitHUB repositories available at https://archive.ics.uci.edu/ml/datasets/liver+disorders and https://github.com/SanikaVT/Liver-disease-prediction, respectively.
